The article "Enterprise Risk Assessment Based on Machine Learning" was published in 2021. Journal: Comput Intell Neurosci.

# Enterprise Risk Assessment Based on Machine Learning

**DOI:** 10.1155/2021/6049195

**Published:** 2021-11-16

**Authors:** Boning Huang, Junkang Wei, Yuhong Tang, Chang Liu

**Affiliations:** ^1^Shenzhen University Webank Institute of Fintech, Shenzhen University, Shenzhen 518052, China; ^2^School of Pharmaceutical Sciences, Sun Yat-sen University, Guangzhou 510630, China; ^3^School of Business and Tourism, Sichuan Agricultural University, Chengdu 610000, China; ^4^Department of Qualitative Economics and Mathematics, School of Statistics and Mathematics, Zhongnan University of Economics and Law, Wuhan 430073, China

## Abstract

Scientific risk assessment is an important guarantee for the healthy development of an enterprise. With the continuous development and maturity of machine learning technology, it has played an important role in the field of data prediction and risk assessment. This paper conducts research on the application of machine learning technology in enterprise risk assessment. According to the existing literature, this paper uses three machine learning algorithms, i.e., random forest (RF), support vector machine (SVM), and AdaBoost, to evaluate enterprise risk. In the specific implementation, the enterprise's risk assessment indexes are first established, which comprehensively describe the various risks faced by the enterprise through a number of parameters. Then, the three types of machine learning algorithms are trained based on historical data to build a risk assessment model. Finally, for a set of risk indicators obtained under current conditions, the risk index is output through the risk assessment model. In the experiment, some actual data are used to analyze and verify the method, and the results show that the proposed three types of machine learning algorithms can effectively evaluate enterprise risks.

## 1. Introduction

With the development of artificial intelligence and the advent of the era of big data, many scholars have used machine learning methods to conduct extensive research on risk assessment [1–4]. Enterprise risk management plays an important role in the stable operation of financial institutions at home and abroad. The traditional methods of judging whether users are in default can no longer meet the requirements of today's multiple types of data, large number of users, and high risk prediction accuracy [5–7]. A large number of scholars use machine learning methods. In-depth related discussions and a series of research results have been made to prove that the method has good prediction and generalization capabilities [8–10].

In the early days, researchers mainly used risk assessment methods based on statistical learning methods. Methods such as regression analysis were first used in the field of credit risk assessment. The linear discriminant analysis method was used for the credit evaluation system, and a mathematical statistics-based model was built to study the credit risk evaluation problem [11–14]. However, these methods have certain limitations. It is too hypothetical for the data distribution requirements, and the sample classification is based on the variance instead of the mean, so the final classification effect is not particularly strong. Linear regression was used to make a score rating based on the credit status of the lender and actual situation [15–18] to forecast the credit risk of bank customers. In essence, the linear regression method uses the existing user credit data to perform regression prediction on users with unknown credit status and finally obtains the probability of whether the user defaults. However, the linear regression also has certain drawbacks [19–22]. The value range it obtains is between plus and minus infinity, and the emergence of logistic regression has just solved this problem. Wiginton et al. first proposed the logistic regression model for credit evaluation [20]. Logistic regression uses the sigmoid function to convert the value obtained after linear regression into a probability value and sets an empirical threshold between 0 and 1 to realize the binary classification problem [23–25].

The risk assessment model based on machine learning has gradually emerged in recent years, showing its superiority compared with traditional risk assessment methods. Common modern machine learning methods include BP neural network, K nearest neighbors (KNN), support vector machine (SVM), etc. In addition, the machine learning methods based on tree models are also widely used in risk assessment, such as basic decision tree models and integrated models such as random forest (RF), GBDT, XGBoost, and LightGBM. Makowski first used modern machine learning methods for risk assessment, in which the credit data were employed to build a model on the classification tree to classify good and bad customers. KNN was also validated more efficiently for two-class classification problem. The artificial neural network model was applied to the personal credit scoring model, which constructed a scoring system based on user credit data. The experimental results show that ensemble models such as RF perform very good in risk assessment. Some researchers pointed out that the machine learning method is mainly to model the historical risk data through supervised learning. After a series of operations such as data processing and feature extraction, the constructed model is used to predict user behavior and characteristics to determine the enterprise risk.

According to the existing literature, this paper uses machine learning algorithms for enterprise risk assessment. Specifically, three types of representative machine algorithms: RF, SVM, and AdaBoost, are used to analyze and evaluate the risk of a certain company. Based on the establishment of a corporate risk indicator system, three types of machine learning algorithms are trained using corporate historical data to obtain a reliable evaluation model. On this basis, the current state of the enterprise is evaluated and judged, and its risk assessment results are obtained. In the experiment, actual data are used to test and evaluate the performance of the three types of machine learning algorithms, and the results show their effectiveness and reliability.

## 2. Index for Evaluation of Enterprise Risk

The risk status of the enterprise directly determines the borrower's ability and willingness to repay the loan with cash flow. Therefore, it is necessary to establish a scientific and intuitive indicator system to provide support for bank loan decision making, so as to make evaluations scientifically and objectively. For example, in the analysis of factors affecting credit decision making, it should comprehensively consider the various influencing factors of credit risk. According to the previous research studies, this paper uses the seven evaluation indicators to describe the enterprise risk, which are current ratio, quick ratio, inventory turnover ratio, asset-liability ratio, tangible net worth debt ratio, net asset interest rate, and multiples of interest earned. The above indicators are specifically defined as follows:

   *x*1 = current ratio = total current assets/total current liabilities. This index reflects the company's ability to repay short-term debt. The more the current assets and the fewer the short-term debts, the greater the current ratio and the stronger the company's short-term debt repayment ability.
   *x*2 = quick ratio = (total current assets−inventory)/total current liabilities.
   This index can reflect the company's ability to repay short-term debt. Because current assets still include inventories that have a slower realization rate and may have depreciated, the current assets are deducted from inventories and then compared with current liabilities to measure the company's short-term debt solvency.
   *x*3 = inventory turnover rate = product sales cost/[(beginning inventory + ending inventory)/2]. This index is the main indicator of inventory turnover speed. Carrying high inventory turnover rate and shortening the business cycle can improve the company's liquidity.
   *x*4 = asset − liability ratio = (total liabilities/total assets) ×100%. This index reflects the ratio of capital provided by creditors to total capital. This index is also called the debt-to-business ratio.
   *x*5 = tangible net worth debt ratio = [total liabilities/(shareholder equity-net intangible assets)]×100%.
   The extension of the property rights ratio index more cautiously and conservatively reflects the degree to which the capital invested by creditors is protected by shareholders' rights during the liquidation of the enterprise. Regardless of the value of intangible assets, including goodwill, trademarks, patent rights, and nonpatent technologies, they may not be used to repay debts. For the sake of caution, they will all be regarded as insolvent.
   *x*6 = net asset interest rate = net profit/[(total assets at the beginning of the period + total assets at the end of the period)/2] × 100%. This index compares the net profit of the company for a certain period with the company's assets, showing the comprehensive utilization effect of the company's assets. The higher the index, the higher the efficiency of asset utilization, indicating that the company has achieved good results in increasing income and saving funds. Otherwise, the opposite conclusion is true.
   *x*7 = multiple of interest earned = profit before interest and tax/interest expense = (total profit + financial expenses)/(interest expense in financial expenses + capitalized interest).

The ratio of business income to interest expense is used to measure the company's ability to repay the interest on borrowings. It is also called interest protection multiple. As long as the multiple of the interest earned is large enough, the enterprise has sufficient ability to repay the interest.

## 3. Models of Risk Assessment

This paper mainly selects three types of machine learning algorithms: RF, SVM, and AdaBoost, to train enterprise risk assessment models. Their basic principles are introduced as follows [18–24].

### 3.1. RF

RF is one of the most commonly used and most powerful supervised learning algorithms, which takes into account the ability to solve regression and classification problems. Random forest is an algorithm that integrates multiple decision trees through the idea of ensemble learning. For the classification problems, the output category is determined by the mode of individual tree output. In the regression problem, the output of each decision tree is averaged to get the final regression result. The specific steps of the RF algorithm are as follows:

(1) The bootstrap resampling method is applied to randomly sample *s* subtraining sets with replacement in the original dataset to form *s* decision trees, namely, *D*_1_, *D*_2_, *D*_3_..., *D*_*s*_. The *s* value is selected according to the stability of the error curve of the model.
(2) The number *m* of preselected variables of the tree node is specified, that is, *m* variables are randomly generated for the construction of the binary tree on the node. The *m* value is selected by successively calculating the residual sum of squares of the model, so that the *m* value with the smallest residual sum of squares is the optimal number of variables.
(3) For a single decision tree, the nodes are recursively partitioned according to the principle of minimum node impurity (that is, the Gini coefficient is the smallest) among the *m* variables. The Gini coefficient is defined as follows:
  (1) $$\begin{array}{c} \text{Gini}\left(t\right)=1-\sum_{j}{\left[p\left(j|t\right)\right]}^{2}, \end{array}$$
 where *t* is a decision tree node and *p*(*j|t*) is the probability of category *j* at node *t*.
(4) Each decision tree is traversed and step (3) is repeated. The decision tree grows arbitrarily without pruning operations.
(5) The *s* decision trees form a forest, and the voting method is used to determine and classify the classified data.

### 3.2. SVM

The basic idea of SVM is to map the data to the high-dimensional feature space through nonlinear mapping and realize the linear regression transformation from the nonlinear function estimation problem to the high-dimensional feature space. The training samples are denoted as (*x*_*i*_, *y*_*i*_), *i*=1,2, ⋯, *N*, *x*_*i*_ ∈ *R*^*n*^ is the input vector, *y*_*i*_ ∈ *R* is the corresponding output value, and, *N* is the number of training samples. The linear model of the high-dimensional space can be expressed as follows:

(2) $$\begin{array}{c} f\left(x,\omega \right)=\sum_{j=1}^{m}\omega_{j}\Phi {\left(x\right)}_{j}+b, \end{array}$$

where *x* is the input vector; *ω* is the feature space coefficient vector; Φ(*x*)_*j*_, *j*=1,2, ⋯, *m*, is the nonlinear transfer function; *ω*_*j*_(*j*=1,2, ⋯, *m*) is the coefficient of the corresponding Φ(*x*)_*j*_ feature space; and *b* is the deviation term of the high-dimensional space. The structural risk function *R*(*ω*) is constructed as follows:

(3) $$\begin{array}{c} R\left(\omega \right)=\frac{1}{2}\omega^{2}+C\sum_{i=1}^{N}L_{\varepsilon }\left(y_{i},f\left(x_{i},\omega \right)\right), \end{array}$$

where ‖*ω*‖ is the Euclidean distance of the feature space coefficient vector; *C* is the penalty coefficient; and *L*_*ε*_(*y*_*i*_, *f*(*x*_*i*_, *ω*)) is the loss function, in which *y*_*i*_(*i*=1,2, ⋯, *N*) is the sample output value and *f*(*x*_*i*_, *ω*)(*i*=1,2, ⋯, *N*) is the output value of the corresponding *x*_*i*_ in high-dimensional space.

This paper uses a linear insensitive loss function, which is defined as follows:

(4) $$\begin{array}{c} L_{\varepsilon }\left(y_{i},f\left(x_{i},\omega \right)\right)=\left\{\begin{array}{cc} 0, & \left|f\left(x,\omega \right)-y\right|<\varepsilon ,\\ \left|f\left(x,\omega \right)-y\right|-\varepsilon , & \left|f\left(x,\omega \right)-y\right|>\varepsilon . \end{array}\right. \end{array}$$

In order to minimize the structural risk function *R*(*ω*), the regression equation can be written as

(5) $$\begin{array}{c} f\left(x\right)=\sum_{i=1}^{N}\left(\alpha_{i}-\alpha_{i}^{*}\right)K\left(x_{i},x\right)+b,\\ \sum_{i=1}^{N}\left(\alpha_{i}-\alpha_{i}^{*}\right)=0,\;\alpha_{i},\alpha_{i}^{*}\in \left[0,C\right], \end{array}$$

where *α*_*i*_ and *α*_*i*_^*∗*^ are the Lagrangian multipliers, which can be solved by the minimum optimization algorithm of the dual problem sequence, and the kernel function *K* is defined as the inner product of the eigenvectors after nonlinear transformation, i.e.,

(6) $$\begin{array}{c} K\left(x_{i},x\right)=\langle \Phi \left(x_{i}\right),\Phi \left(x\right)\rangle . \end{array}$$

Any function that satisfies Mercer's condition can be used as a kernel function. If the kernel function coefficient corresponding to a sampling point is not zero, then the sampling point is a support vector. The commonly used kernel functions in SVM include Gaussian kernel function, radial basis kernel function, etc.

### 3.3. AdaBoost

This paper is based on single-label multi-class problems, so we choose the simpler and direct AdaBoost algorithm. The main steps of the algorithm are as follows:

(1) The weight distribution of training data points is initialized. The weak learner iteratively operates *T* times and produces a weak hypothesis *h* : *X*⟶*Y* after each iteration. The *T* value can be selected according to the error curve of the final strong classification.
(2) The calculation of classification error rate is performed using the following formula:
  (7) $$\begin{array}{c} h_{t}\;:\xi_{t}=\sum_{i:h_{t}\left(x_{i}\right)\neq y_{i}}D_{t}\left(i\right), \end{array}$$
 where *D*_*t*_ is the weight distribution of the training data at the *t*th iteration. In each iteration, if *ξ*_*t*_ > 1/2, then this iteration will be aborted.
(3) The weight is assigned to the weak hypothesis according to the classification error rate, and the weight distribution of training data points is updated as follows:
  (8) $$\begin{array}{c} D_{t+1}\left(i\right)=\frac{D_{t}\left(i\right)}{Z_{t}}\times \left\{\begin{array}{c} \beta_{t}\;h_{t}\left(x_{i}\right)=y_{i}\\ 1\text{ others} \end{array}\right., \end{array}$$
where *β*_*t*_=*ξ*_*t*_/(1 − *ξ*_*t*_) and *Z*_*t*_ is the normalization constant.
(4) All the weak hypotheses with weights are combined into the final prediction function. The calculation formula is as follows:
  (9) $$\begin{array}{c} h_{\text{fin}}\left(x\right)=\underset{y\in Y}{\arg\max}\sum_{t=1}^{T}\ln\left(\frac{1}{\beta_{t}}\right)\left[h_{t}\left(x\right)=y\right]. \end{array}$$

The basic idea of the method in this paper is described in Figure 1. Based on the historical training data, the indicator feature vector is constructed according to the method described in Section 2. Accordingly, three types of machine learning algorithms are trained to obtain evaluation models. In the test phase, for the acquired data, the index feature vector is also constructed, and the training evaluation model is input to obtain the current enterprise's risk evaluation result.

## 4. Experiments and Analysis

### 4.1. Dataset and Evaluation Indicators

The data sample used in this paper is to select 300 loan companies from a bank and divide them into two categories, i.e., “performance companies (*y*=1)” and “default companies (*y*=−1)” according to their financial status, operating status, and past credit records. According to the established safety evaluation index system, each sample is a 7-dimensional vector. First of all, the sample data are processed for robustness and efficiency. In view of the large sample data volume and the smoothness of the data, the double triple standard deviation test is used to eliminate abnormal data, and the total number of effective samples is finally obtained as 500. Among them, 255 companies are able to repay bank credit loans, and the remaining 245 are unable to repay loans on time.

In order to quantitatively analyze the performance of the proposed method, this paper selects accuracy and ROC curve as evaluation indicators. Among them, the accuracy index is a simple and effective index for evaluating classification and prediction performance and refers to the proportion of the correct evaluation samples in the total samples. Area under the curve (AUC) can measure the posterior probability, classification performance, and ranking performance of machine learning algorithms, so it has been widely used in the field of machine learning algorithms. Taking false positive class rate (FPR) as the horizontal axis and true positive class rate (TPR) as the vertical axis, a set of different (FPR, TPR) points can be obtained on the coordinate axis by continuously adjusting the classifier threshold. These points are connected into a line to get the ROC curve of the classifier. The ROC curve cannot be directly used as the evaluation index of the classifier, and the AUC value is generally used as the quantitative criterion.

## 5. Result and Analysis

This paper uses K-fold cross validation. Generally, K is 10 because it has relatively low bias and variance. Therefore, this paper divides 500 corporate risk data into 10 equal parts, namely, T1, T2, T3,..., T10. Take T*i* as the test dataset, and the remaining part is the training dataset, thereby constructing the *i*th group of test training sets (Test*i*, Train*i*) (*i* = 1, 2, ..., 10). The average of the accuracy value and AUC value of each model is calculated, and the statistical results are shown in Table 1.

The following can be seen from Table 1. (1) Combining the two evaluation index standards, the SVM model is effective, and the RF and AdaBoost models have excellent performance. (2) From the perspective of accuracy, the AdaBoost model is better than the SVM and RF models; from the perspective of the AUC value, the RF model is almost the same as the AdaBoost model, and both are better than the SVM model.

Considering the two evaluation indicators, the accuracy value of the AdaBoost model is 1.2% higher than that of the RF model, and the AUC value is higher than that of the RF model. The relationship between enterprise risk levels is slightly better than SVM and RF models.

Taking into account the possible noise impact of actual data, this paper applies different degrees of noise conditions to 500 sample data and uses signal-to-noise ratio (SNR) to measure the noise level.  Figure 2 shows the accuracy performance curves of the three methods under different SNRs. It can be seen from the comparison that the noise robustness of the RF and AdaBoost methods is still better than that of the SVM method, reflecting its stronger robustness.

## 6. Conclusion

Statistical learning methods are widely used in risk assessment due to their simple structure and strong interpretation. However, based on the assumption that there is a linear relationship between variables, the prediction effect lacks accuracy and cannot fully reflect the risk status in many cases. The risk assessment model constructed by modern machine learning methods has high accuracy through data training and has broad application prospects in enterprise risk assessment. In this paper, three machine learning algorithms of RF, SVM, and AdaBoost are applied to enterprise risk assessment, which are verified based on actual data. The comparison shows that RF and AdaBoost have higher accuracy in predicting risk. Different machine learning methods have different advantages. Combining different machine learning methods or using integrated learning methods for data feature processing, the performance of the proposed method can be further improved.

## Figures and Tables

**Figure 1:** Basic procedure of the proposed method.

**Figure 2:** Accuracy of the three machine learning algorithms.

**Table 1:** Comparison of performance of the three machine learning algorithms.

	Accuracy (%)	AUC
RF	87.9	0.861
SVM	85.2	0.837
AdaBoost	90.1	0.878

## Data Availability

The dataset can be accessed upon request.
